# Causal relationship between nutritional assessment phenotypes and heart failure: A Mendelian randomization study

**DOI:** 10.1016/j.heliyon.2024.e28619

**Published:** 2024-03-26

**Authors:** Yun-Hu Chen, Mo-Qing Yin, Li-Hua Fan, Xue-Chun Jiang, Hong-Feng Xu, Xing-Yu Zhu, Tao Zhang

**Affiliations:** a Cardiovascular Department, Taicang TCM Hospital Affiliated to Nanjing University of Chinese Medicine, Suzhou, 215400, China; b Clinical Pharmacy Department, Taicang TCM Hospital Affiliated to Nanjing University of Chinese Medicine, Suzhou, 215400, China; c Cardiovascular Department, Changzhou Hospital Affiliated to Nanjing University of Chinese Medicine, Changzhou, 213003, China

**Keywords:** Mendelian randomization, Causal association, Nutritional assessment, Heart failure, Risk factors, Educational attainment, Mediation analysis

## Abstract

**Introduction:**

Malnutrition is strongly associated with heart failure (HF); however, the causal link remains unclear. We used Mendelian randomization (MR) to infer causal associations between different nutritional assessment phenotypes and HF and to analyze whether these associations were mediated by common HF risk factors.

**Methods:**

Two-sample bidirectional MR was used to infer causal associations between nutritional assessment phenotypes and HF. Mutual influences between different nutritional assessment phenotypes and potential correlations were estimated using multivariate MR methods. Two-step MR was used to quantify the mediating effects of common HF risk factors on the causal associations.

**Results:**

Three phenotypes were positively associated with the development of HF: waist circumference (WC) (odds ratio [OR] = 1.74; 95% confidence interval [CI], 1.60–1.90; *P* = 3.95 × 10^−39^), body mass index (BMI) (OR = 1.70; 95%CI, 1.60–1.80; *P* = 1.35 × 10^−73^), and whole body fat mass (WBFM) (OR = 1.54; 95%CI, 1.44–1.65; *P* = 4.82 × 10^−37^). Multivariate MR indicated that WBFM remained positively associated with HF after conditioning on BMI and WC (OR = 2.05; 95%CI, 1.27–3.31; *P* = 0.003). Three phenotypes were negatively correlated with the development of HF: usual walking pace (UWP) (OR = 0.40; 95%CI, 0.27–0.60; *P* = 8.41 × 10^−6^), educational attainment (EA) (OR = 0.73; 95%CI, 0.67–0.79; *P* = 2.27 × 10^−13^), and total cholesterol (TC) (OR = 0.90; 95%CI, 0.84–0.96; *P* = 4.22 × 10^−3^). There was a bidirectional causality between HF and UWP (Effect estimate = −0.03; 95%CI, −0.05 to −0.01; *P* = 1.95 × 10^−3^). Mediation analysis showed that common risk factors for HF (hypertension, coronary artery disease, cardiomyopathy, and valvular heart disease) mediated these causal associations (all *P* < 0.05).

**Conclusions:**

BMI, WC, and WBFM are potential risk factors for HF, and the correlation between WBFM and HF was significantly stronger than that between BMI and WC, and HF. EA, UWP, and TC are potential protective factors against HF. Common risk factors for HF mediate these causal pathways. Early identification of potential risk or protective factors for HF patients from the dimension of nutritional status is expected to further improve patient outcomes.

## 1 Introduction

Despite substantial advancements in heart failure (HF) treatment in recent years, the disease remains associated with significant morbidity and mortality rates. The prevalence of HF in the general adult population of industrialized countries has been reported to be between 1% and 3%, with a mortality risk of 15%–30% at 1 year and up to 75% at 5 years in specific HF populations [1]. Malnutrition typically refers to a state of energy or nutrient deficiency resulting from inadequate intake or impaired utilization [2,3]. Depending on the various malnutrition assessment methods used, the prevalence of malnutrition in patients with HF is estimated to range between 15% and 90% [[4], [5], [6]]. Furthermore, patients who are moderately to severely malnourished face a 6- to 10-fold higher risk of death than those without malnutrition [7]. Nutritional status has garnered increasing attention as a variable factor and a potential target for the prevention and intervention of HF.

Malnutrition or the risk of malnutrition is strongly associated with clinical outcomes in patients with HF. However, epidemiological studies have produced inconsistent or even contradictory results regarding the role of specific phenotypes of nutritional assessment such as cholesterol, in the development of HF. Additionally, it is intuitive that HF and malnutrition may cause one another. Malnutrition may aggravate underlying cardiac dysfunction due to cytokines produced by metabolic abnormalities, and HF may also lead to malnutrition due to multiple complications, psychological disorders, loss of appetite, etc [8]. Notably, that these existing pieces of evidence are mainly from traditional observational studies, and the possibility of confounding and reverse causality cannot be completely excluded. Therefore, these conclusions should be interpreted with caution. Whether there is a causal association between different nutritional assessment phenotypes and the onset of HF is unclear.

Mendelian randomization (MR) is an emerging tool in genetic epidemiology that uses genetic variants to assess the causal associations between exposure and outcome [9,10]. Because genetic variation is randomly assigned before conception and does not change at will, MR largely overcomes the inherent shortcomings of traditional observational studies and can more accurately observe causal relationships between variables. To the best of our knowledge, no MR studies have inferred a potential causal relationship between different nutritional assessment phenotypes and HF. Here, we conducted an MR study based on currently publicly accessible genome-wide association study (GWAS) datasets to genetically infer causal effects between different nutritional assessment phenotypes (anthropometric measurements, biochemical analysis, clinical evaluation, and environment) and HF and to analyze whether these associations were mediated by common HF risk factors.

## 2 Materials and methods

### 2.1 MR study design

This study used a two-sample, bidirectional, multivariate, two-step MR design that complied with the STROBE-MR statement [11].

Single nucleotide polymorphisms (SNPs) strongly associated with exposures (different nutritional assessment phenotypes) were used as genetic instrumental variables to infer causality between exposures and outcome (HF). Exposures and outcome were interchanged to perform reverse MR and verify the presence or absence of reverse causality. Mutual influences between different nutritional assessment phenotypes and potential correlations were estimated using multivariate MR methods. Two-step MR was used to quantify the mediating effects of common HF risk factors on the causal associations.

The MR design had to satisfy three assumptions (Fig. 1): (i) association assumption: SNPs are highly associated with predicted exposures (*P*＜5 × 10^−8^), (ii) independence assumption: SNPs are independent of known potential confounders, and (iii) exclusivity assumption: SNPs influence the outcome through exposure factors and are not directly related to the outcome.

**Fig. 1:** Three assumptions of the MR analysis. The red crosses in the figure indicate that the assumptions are not allowed. SNP, Single nucleotide polymorphism; MR, Mendelian randomization.

Summary data used in this study were obtained from publicly available GWAS_s_ of European ancestry. The relevant cohort ethics committees for human studies approved these data; therefore, separate ethical approval was not required for this study.

### 2.2 GWAS summary data for nutritional assessment phenotypes

Ten commonly used and easily available nutritional assessment phenotypes were used as exposure factors, including body mass index (BMI), whole body fat mass (WBFM), waist circumference (WC), hemoglobin, albumin, total cholesterol (TC), vitamin D, usual walking pace (UWP), right hand grip strength, and educational attainment (EA) (Table 1). The GWASs for these phenotypes were obtained from the Genetic Investigation of ANthropometric Traits (GIANT), UK Biobank Round 2, FinnGen, and the Social Science Genetic Association Consortium (SSGAC). The GIANT consortium is an international collaboration that aims to identify the genetic loci that regulate human size and shape, including measures of height and adiposity. The UK Biobank, a large biomedical database and research resource, contains genetic and health information from half a million UK participants. FinnGen is a project designed to collect and analyze genomic and health data from half a million Finnish biobank participants. The GWAS for EA was derived from a study published by Lee and colleagues [12].

**Table 1:** GWAS details of nutritional assessment phenotypes and HF.

Traits	Introduction to Traits	Value Type	Consortium	Sample Size	Ancestry
Body Mass Index	Weight/height^2^	Continuous,kg/m^2^	GIANT	681,275	European
Waist circumference	In the standing position, the length measured horizontally with a tape measure at the narrowest point of the waist.	Continuous, cm	UK BIOBANK	500,290	European
Whole body fat mass	Body composition estimation by impedance measurement. Total fat mass in Kg, in 0.1 Kg increments.	Continuous, Kg	UK BIOBANK	492,256	European
Albumin (quantile)	Blood biochemistry Biomarker, Measured by BCG analysis on a Beckman Coulter AU5800	Continuous, g/L	UK BIOBANK	432,221	European
Haemoglobin concentration	Blood biochemistry Biomarker, Result of "Haemoglobin Concentration" assay, performed on blood sample, obtained from UK Biobank assessment centre visit.	Continuous, grams/decilitre	UK BIOBANK	479,219	European
Cholesterol (quantile)	Blood biochemistry Biomarker, Measured by CHO-POD analysis on a Beckman Coulter AU5800.	Continuous, mmol/L	UK BIOBANK	470,716	European
Vitamin D deficiency	Diagnosed according to ICD-10 Version:2016 E55.	Binary	FinnGen	355238	European
Usual walking pace	ACE touchscreen question "How would you describe your usual walking pace? " Slow pace is defined as less than 3 miles per hour. Steady average pace is defined as between 3 and 4 miles per hour. Fast pace is defined as more than 4 miles per hour.	Categorical (single)	UK BIOBANK	499,626	European
Hand grip strength (right)	Measured using a dynamometer for at least 3 s, and the maximum grip strength was read in whole kilogram force units.	Integer, Kg	UK BIOBANK	499,280	European
Educational attainment	Measured as the number of years of schooling that individuals completed.	Continuous, Year	Social Science Genetic Association Consortium (SSGAC)	1,131,881	European
Heart failure	Details of the definitions used to determine heart failure status in each study are provided in the Supplementary data from the GWAS original article (PMID: 31919418).	Binary	HERMES	977,323	European

GWAS, Genome-wide association study; HF, Heart failure.

### 2.3 GWAS summary data for HF

GWAS summary statistics for HF were derived from the HEart failure Molecular Epidemiology for Therapeutic targetS (HERMES) consortium (Table 1). The original article is available on the Cardiovascular Disease Knowledge Portal (CVDKP) (https://cvd.hugeamp.org/downloads.html). Shah and colleagues conducted a GWAS of 47,309 cases and 930,014 controls of European ancestry from 26 studies of the HERMES consortium [13]. The study samples included population-based cohorts (17 studies, 38,780 HF cases, 89,657 controls) and case-control samples (nine studies, 8529 cases, 36,357 controls). A meta-analysis using fixed-effects inverse variance weighted (IVW) linked 8,281,262 common and low-frequency variants to HF risk was performed. Finally, 12 independent SNPs were found at 11 loci that were significantly associated with HF, including 10 loci that have not been previously reported to be associated with HF.

### 2.4 Selection and validation of SNPs

SNPs closely associated with nutritional assessment phenotypes were selected with a genome-wide significance threshold of *P* < 5 × 10^−8^, and the threshold was relaxed to *P* < 5 × 10^−6^ if there were insufficient SNPs for the final MR analysis. The distribution of genetic variation may not be random because of nonrandom correlations (linkage disequilibrium) between two or more genes, which may obscure or misrepresent causal associations. Linkage disequilibrium was removed by setting the parameters (r^2^ = 0.001 and kb = 10,000). When a small number (<10% in this study) of SNPs in the exposure were unrecognizable in the outcome, the proxy SNP was not used, and MR analysis was continued. If >10% of the SNPs were unrecognizable in the outcome, replacement of the exposed GWAS summary data was considered. In addition, to prevent any bias introduced by weak instrumental variables, we calculated the F-statistics for the screened SNPs. The larger the F value, the more accurate the causal inference; weak instrumental variables with an F value < 10 were excluded. The formula for calculating F-value is as follows [14]:

$$F‐\text{value}=\frac{N-k-1}{k}\times \frac{R^{2}}{{1-R}^{2}}$$

$$R^{2}=2\times \left(1‐\text{MAF}\right)\times \text{MAF}\times \beta^{2}$$

Note: N: number of samples of exposure GWAS; k: number of instrumental variables; R^2^: the extent to which the instrumental variable explains exposure.; MAF: minor allele frequency; β: effect size of SNP on exposure.

When genetic variants affect the development of HF through a pathway other than "genetic variant-nutritional assessment phenotype-HF," the genetic variants are considered pleiotropic, which violates the basic assumptions of MR. SNPs with *P* < 5 × 10^−5^ in the outcome GWAS dataset were excluded to fulfill the exclusivity assumption and prevent pleiotropy.

### 2.5 MR analysis

We investigated the causal relationship between nutritional assessment phenotypes and HF using the IVW method, which is one of the most commonly used MR analysis methods. IVW provides efficient statistical efficacy by assuming that all variables are valid, disregarding the presence of intercept terms in the analysis, and using the inverse of the variance of the outcomes as fitting weights [15]. The weighted median and MR-Egger were used as supplements for IVW analysis. The weighted median is an MR analysis method based on the median principle that provides valid estimates if more than 50% of the information comes from valid instrumental variables [16]. The MR-Egger method also uses the inverse of the variance of the outcomes as weights for fitting; however the regression considers the presence of an intercept term so that directional pleiotropy can be quantified and interpreted to provide unbiased estimates [17]. The purpose of using multiple MR methods is to provide more robust estimates for the MR analyses. To reduce the probability of type II errors (false negatives) and to improve the accuracy and reliability of the results of the MR analyses, we further calculated the statistical power, where a higher power indicates a lower probability of committing a type II error and a greater degree of confidence that the results are significant.

Additionally, we performed a sensitivity analysis of the MR analysis results. Heterogeneity among the SNPs used for MR analysis was assessed using the IVW Cochran's Q statistic [16]. Fixed-effect IVW models were used when no heterogeneity between SNPs was detected; otherwise, random-effect IVW models were used to mitigate the effect of heterogeneity on the MR analysis [18].

Leave-one-out analysis helped determine whether the overall estimate was disproportionately affected by individual SNPs. MR-Egger intercept analysis detected the presence of horizontal pleiotropy, which, if the intercept was not zero (*P* < 0.05), suggested that the outcome was present when the exposure did not produce an effect. In addition, the Mendelian Randomization Pleiotropy RESidual Sum and Outlier (MR-PRESSO) was used to detect outliers and correct for possible heterogeneity and pleiotropy [19,20].

Multivariate MR analysis was performed on different nutritional assessment phenotypes with potential correlations to jointly explore their association with outcomes. Multivariate MR analyses required that each exposure was associated with at least one genetic variant. The two-step MR method was used for mediation analysis, and the coefficient product method was used to calculate and test the mediation proportion and confidence interval [21,22].

Because of multiple tests between the two samples, the Bonferroni method was used to correct the significance threshold.

All statistical analyses were performed using the "TwoSampleMR 0.5.7″, "MRPRESSO 1.0″ and "MendelianRandomization 0.7.0″ packages in R version 4.3.0.

The two-sample MR analysis process designed for this study is illustrated in Fig. 2.

**Fig. 2:** Flow chart of the MR analysis process designed for this study. Exposures and outcome were interchanged when reverse-MR analyses were performed.

## 3 Results

### 3.1 Instrumental variables

We screened a certain number of SNPs from each of 10 nutritional assessment phenotypes (BMI, WBFM, WC, hemoglobin, albumin, TC, vitamin D deficiency, UWP, right hand grip strength, and EA) for the genetic prediction of HF development. These SNPs of different phenotypes explained 0.16–19.2% of the variance in exposure, and the F-value for individual SNPs was greater than 10, suggesting that these SNPs were robust and feasible for assessing causality (Table 2).

**Table 2:** Genetic instrumental variables.

Traits	*P*	No. of SNPs	R^2^	F_min_	Traits	*P*	No. of SNPs	R^2^	F_min_
BMI	<5 × 10^−8^	503（510-7）	4.92%	26.73	Vitamin D deficiency	<5 × 10^−6^	8（-0）	19.21%	3571.11
WC	<5 × 10^−8^	257(260-3)	2.76%	31.69	TC	<5 × 10^−8^	153(160-7)	5.80%	37.61
WBFM	<5 × 10^−8^	304（307-3）	4.28%	38.81	UWP	<5 × 10^−8^	42(44-2)	0.16%	14.99
Albumin (quantile)	<5 × 10^−8^	193(195-2)	4.77%	39.27	Hand grip strength (right)	<5 × 10^−8^	123(123-0)	0.75%	19.84
Haemoglobin concentration	<5 × 10^−8^	274(277-3)	4.06%	25.45	EA	<5 × 10^−8^	314(316-2)	2.23%	27.92

Note: The number of SNPs in parentheses is the number of SNPs screened minus the number of SNPs associated with HF. SNP, Single nucleotide polymorphism; BMI, Body mass index; WC, Waist circumference; WBFM, Whole body fat mass; TC, Total cholesterol; UWP, Usual walking pace; EA, Educational attainment.

### 3.2 Results of MR analysis

We assessed the causal relationship between nutritional assessment phenotypes and HF using three algorithms (MR-Egger, weighted median, and IVW), with the IVW approach being predominant.

The IVW analysis revealed causal associations between the six nutritional assessment phenotypes and HF, and all had a statistical power of 1. Three of these phenotypes were positively associated with the development of HF, with the risk of development being, in descending order, WC (odds ratio [OR] = 1.74; 95% confidence interval [CI], 1.60–1.90; *P* = 3.95 × 10^−39^), BMI (OR = 1.70; 95%CI, 1.60–1.80; *P* = 1.35 × 10^−73^), and WBFM (OR = 1.54; 95%CI, 1.44–1.65; *P* = 4.82 × 10^−37^). Due to the potential correlation of these three phenotypes with HF, we further evaluated the interactions among them using multivariate MR methods. In the IVW multivariate model, after adjustment, BMI was not significantly associated with the occurrence of HF (*P* = 0.439), while WC was negatively associated with HF (OR = 0.52; 95%CI, 0.30–0.90; *P* = 0.021) and WBFM was positively correlated with HF (OR = 2.05; 95%CI, 1.27–3.31; *P* = 0.003). The other three phenotypes were negatively correlated with HF development, suggesting a protective effect against HF development. The protective effects were, in descending order, UWP (OR = 0.40; 95%CI, 0.27–0.60; *P* = 8.41 × 10^−6^), EA (OR = 0.73; 95%CI, 0.67–0.79; *P* = 2.27 × 10^−13^), and TC (OR = 0.90; 95%CI, 0.84–0.96; *P* = 4.22 × 10^−3^). The weighted median and MR-Egger analyses for some of the phenotypes in the above analyses, although not significant, still showed effect sizes that were consistent with the direction of IVW and thus were still considered evidence of a causal association.

It is worth mentioning that although IVW analysis showed a negative association of albumin with the development of HF (OR = 0.90; 95% CI, 0.84–0.96; *P* = 4.22 × 10^−3^), MR-Egger and weighted madian showed effect values opposite to the IVW, and in addition the Egger's intercept test showed the presence of pleiotropy (*P* = 0.019), which violated the assumptions of MR. We excluded two SNPs (rs3184504, rs4970834) that were highly correlated with HF, and also excluded the outliers using MR-PRESSO, which still failed to avoid pleiotropy when MR analysis was performed again. Therefore, it is not yet possible to confirm whether there is a causal association between albumin levels and HF.

In contrast, no positive causal association was observed between the remaining assessment phenotypes (hemoglobin level, vitamin D deficiency, and hand grip strength) and the development of HF. Overall, these results suggest that from a genetic perspective, BMI, WBFM, and WC may increase the risk of HF development and are risk factors for HF, whereas UWP, EA, and TC reduce the risk of and are protective factors against HF development (Fig. 3, Fig. 4).

**Fig. 3:** Scatter plots of the results of MR analysis of BMI, WC, WBFM, UWP, EA and TC with HF. The horizontal axis represents the impact of SNPs on the exposure, while the vertical axis shows their effect on the outcome. The figure features three lines, each colored differently, to depict the linear regression from the three distinct MR analyses. In panels A, B, and C, ascending lines suggest that the exposure acts as a risk factor for the outcome. Conversely, descending lines in panels D, E, and F imply the exposure serves as a protective factor against the outcome. SNP, Single nucleotide polymorphism; HF, Heart failure; BMI, Body mass index; WC, Waist circumference; WBFM, Whole body fat mass; TC, Total cholesterol; UWP, Usual walking pace; EA, Educational attainment.

**Fig. 4:** Forest plot of the results of the MR analysis. IVW, Inverse variance weighted; MR, Mendelian randomization; HF, Heart failure.

### 3.3 Sensitivity analysis

No evidence of pleiotropy was detected using MR-Egger intercept analysis, except for albumin. Leave-one-out sensitivity analysis showed that the overall estimate was not disproportionately affected by the individual SNP. Funnel plots showed an essentially left-right symmetric distribution of SNPs, indicating no evidence of horizontal pleiotropy.

### 3.4 Reverse MR analysis

To further determine whether there was an inverse causal association between nutritional assessment phenotypes and HF, we repeated the complete MR analysis described above with HF as the exposure and the 10 nutritional assessment phenotypes as the outcomes. Finally, we selected 12 SNPs from the HF GWAS as genetic variables for analysis using the MR-Egger, weighted median, and IVW methods. IVW showed a negative association between HF and UWP (Effect Estimate = −0.03; 95%CI, −0.05 to −0.01; *P* = 1.95 × 10^−3^). Weighted median and MR-Egger analyses showed effect values consistent with IVW, and there was no pleiotropy in the Egger intercept analysis (*P* = 0.940), providing evidence of a causal association. Therefore, the development of HF can lead to a reduction in the UWP.

IVW analysis also showed a positive association between HF and vitamin D deficiency (OR = 3.39; 95%CI, 1.44–7.95; *P* = 4.91 × 10^−3^), but the effect value of the MR-Egger analysis was not consistent with IVW, suggesting that the IVW results were not robust. Thus, HF cannot yet be considered a risk factor for vitamin D deficiency. None of the remaining eight phenotypes in the IVW analysis showed reverse or bidirectional causal associations with HF.

### 3.5 Analysis of mediation

The above MR analysis revealed a causal relationship between the genetically predicted nutritional assessment phenotypes (WC, BMI, WBFM, UWP, EA, and TC) and HF. To further explore whether these causal associations were mediated by known common risk factors of HF (hypertension, coronary heart disease, cardiomyopathy, and valvular heart disease), we performed a mediation analysis using a two-step MR method. To avoid sample overlap, GWAS summary data on risk factors for HF were obtained from the Finnish DF9 database.

Evidence of a positive causal association between hypertension, coronary heart disease, cardiomyopathy, and valvular heart disease, and HF was obtained using two-sample MR, which was consistent with the results of observational studies. Further mediation analysis using the two-step MR method showed that these common HF risk factors mediated the six causal associations. Specifically, hypertension, coronary heart disease, valvular heart disease, and cardiomyopathy simultaneously mediated the causal association of BMI and WC with HF; hypertension, coronary heart disease, and cardiomyopathy mediated the causal associations between WBFM and HF; valvular heart disease mediated the causal associations between TC and HF; hypertension, and coronary heart disease mediated the causal associations between EA and HF; and hypertension mediated the causal associations between UWP and HF (Fig. 5). The mediating effects, percentages of indirect effects, and confidence intervals are presented in Table 3. Significance tests were conducted using the product of coefficients method, and the statistical Z-value of all mediation analyses was >1.96, with a *P*-value of <0.05, suggesting that the mediating effect was significant.

**Fig. 5:** The schematic diagram of the mediation analysis results. "-" represents causal association between exposure and outcome. BMI, Body mass index; WC, Waist circumference; WBFM, Whole body fat mass; TC, Total cholesterol; UWP, Usual walking pace; EA, Educational attainment; HTN, Hypertension; CHD, Coronary heart disease; VHD, Valvular heart disease; CMP, Cardiomyopathy; HF, Heart failure.

**Table 3:** Analysis of intermediation effects.

Exposure	Mediation	Two-sample MR				Analysis of mediation		
		Exposure-mediation		Mediation-outcome (HF)		Mediation effect	Indirect effect (95%CI)	*P*
		OR(95%CI)	*P*	OR(95%CI)	*P*			
BMI	HTN	1.76(1.65–1.87)	9.44 × 10^−74^	1.24(1.20–1.29)	7.26 × 10^−33^	0.125	23.55%(21.24%–25.86%)	2.10 × 10^−24^
BMI	CHD	1.31(1.24–1.42)	2.38 × 10^−16^	1.30(1.23–1.38)	1.40 × 10^−21^	0.077	14.46%(12.17%–16.74%)	2.47 × 10^−10^
BMI	VHD	1.11(1.03–1.21)	4.84 × 10^−3^	1.49(1.34–1.66)	1.31 × 10^−13^	0.045	8.46%(5.30%–11.62%)	7.37 × 10^−3^
BMI	CMP	1.39(1.22–1.58)	3.46 × 10^−7^	1.27(1.13–1.43)	3.01 × 10^−5^	0.081	15.39%(10.63%–20.15%)	1.22 × 10^−3^
WC	HTN	1.79(1.62–1.99)	2.49 × 10^−28^	1.24(1.20–1.29)	7.26 × 10^−33^	0.129	23.20%(20.38%–26.02%)	1.97 × 10^−16^
WC	CHD	1.36(1.23–1.49)	2.12 × 10^−10^	1.30(1.23–1.38)	1.40 × 10^−21^	0.082	14.80%(12.04%–17.59%)	9.50 × 10^−8^
WC	VHD	1.14(1.02–1.27)	1.72 × 10^−2^	1.49(1.34–1.66)	1.31 × 10^−13^	0.053	9.49%(5.33%–13.64%)	2.23 × 10^−2^
WC	CMP	1.34(1.12–1.60)	1.11 × 10^−3^	1.27(1.13–1.43)	3.01 × 10^−5^	0.072	13.02%(7.94%–18.10%)	1.03 × 10^−2^
WBFM	HTN	1.52(1.40–1.64)	1.14 × 10^−25^	1.24(1.20–1.29)	7.26 × 10^−33^	0.093	21.43%(18.75%–24.12%)	1.34 × 10^−15^
WBFM	CHD	1.23(1.13–1.33)	3.00 × 10^−7^	1.30(1.23–1.38)	1.40 × 10^−21^	0.056	13.07%(10.19%–15.96%)	5.72 × 10^−6^
WBFM	CMP	1.28(1.11–1.46)	3.50 × 10^−4^	1.27(1.13–1.43)	3.01 × 10^−5^	0.061	14.05%(8.89%–19.22%)	6.48 × 10^−3^
TC	VHD	0.80(0.72–0.88)	2.96 × 10^−5^	1.49(1.34–1.66)	1.31 × 10^−13^	−0.089	81.13%(65.11%–97.14%)	4.04 × 10^−7^
EA	HTN	0.64(0.58–0.70)	1.23 × 10^−19^	1.24(1.20–1.29)	7.26 × 10^−33^	−0.097	31.30%(29.05%–33.55%)	4.67 × 10^−44^
EA	CHD	0.71(0.64–0.79)	5.31 × 10^−11^	1.30(1.23–1.38)	1.40 × 10^−21^	−0.090	28.88%(25.67%–32.09%)	2.23 × 10^−19^
UWP	HTN	0.31(0.19–0.52)	9.10 × 10^−6^	1.24(1.20–1.29)	7.26 × 10^−33^	−0.252	27.99%(22.13%–33.86%)	1.78 × 10^−6^

BMI, Body mass index; WC, Waist circumference; WBFM, Whole body fat mass; TC, Total cholesterol; UWP, Usual walking pace; EA, Educational attainment; HF, Heart failure; HTN, Hypertension; CHD, Coronary heart disease; VHD, Valvular heart disease; CMP, Cardiomyopathy; MR, Mendelian randomization; OR, Odds ratio; CI, Confidence interval.

## 4 Discussion

In our study, we used an MR design to assess the causal relationships between 10 commonly used nutritional assessment phenotypes and HF. The results showed that genetically predicted BMI, WC, and WBFM were positively associated with the development of HF, and EA, UWP, and TC were negatively associated with the development of HF, with bidirectional causality between UWP and HF. These causal associations may be related to mediating factors such as hypertension, coronary heart disease, cardiomyopathy, and valvular heart disease.

Anthropometric assessment has become an important practice for evaluating nutritional risk in patients with HF. BMI has long been a well-recognized metric for nutritional assessment because of its simplicity and established relationships with associated comorbidities. Previous studies have shown that a high BMI is a risk factor for the development of HF and atrial fibrillation, a finding that is consistent with the results of our MR analysis [[23], [24], [25], [26], [27]]. However, there is still the so-called "obesity-survival paradox [[28], [29], [30], [31]]." This concept is highly controversial because of inconsistent research results. The main reason for this paradox is that the BMI calculation ignores body composition and distribution. In our multivariate model, the effect of BMI on HF was not significant, whereas WBFM had the greatest effect on HF incidence. Therefore, the World Health Organization recommends its use only as an imprecise indicator for nutritional assessment [28]. Body composition assessment has been shown to be useful in evaluating the nutritional status of patients in nutritional assessments [32,33]. WBFM can be obtained using a simple and non-invasive bioelectrical impedance analysis (BIA) method, and WC is an easy-to-use indicator of adipose tissue. The WBFM can be divided into subcutaneous fat and visceral adipose tissue (VAT). VAT has been repeatedly shown to increase the risk of cardiovascular diseases such as HF, and a recent MR study of VAT and HF also confirmed this harm at the genetic level [34]. However, there are conflicting views on the association between WBFM and HF, with some studies suggesting that WBFM is associated with the trajectory of HF development, and is a predictor of poor metabolic outcomes. Excess fat mass is associated with an increased risk of death, whereas a defatted body weight reduces the risk of death [35,36]. A recently published prospective cohort study reached the opposite conclusion, that an increased fat mass index was a predictor of favorable prognosis in an elderly population with HF [37]. The relationship between WC and the onset of HF has been largely confirmed, with an increased incidence of HF and an increased risk of death for every 10 cm increase in WC [38]. The present study supports the adverse role of WBFM and WC in the development of HF in terms of genetic prediction and provides preliminary insights into the causal pathways. To the best of our knowledge, no MR analysis of WC, WBFM, and HF has been reported; therefore, this study complements the current research.

TC is a valid biochemical marker of the nutritional status of patients with HF. Cholesterol is a common nutrient in the human diet that performs certain physiological functions in the body. Although lowering TC has been a component of cardiovascular disease risk prediction models, there is still a great deal of controversy regarding TC and the risk of developing HF [39]. A retrospective study conducted by Halldin showed that TC was not associated with the risk of HF later in life in 50-year-old women [40]. In contrast, another retrospective study showed that TC ≥ 240 mg/dL was positively associated with the risk of HF in postmenopausal Japanese women (HR = 1.70，95%CI, 1.04–2.77) [41]. In addition, a prospective cohort study showed that TC > 200 mg/dL in nondiabetic patients with chronic HF was associated with a 64% reduction in the 5-year risk of death [42]. Therefore, the relationship between TC and HF has not been clarified, and completely opposite conclusions are shown. One reason for this may be the nonlinear association between TC and HF, and another may be that TC reflects the underlying nutritional status. Since malnutrition is strongly associated with increased mortality, the impact of malnutrition on disease needs to be considered as well [43]. Our study showed that TC was negatively associated with the development of HF; that is, it was protective against the development of HF, and mediational analyses suggested that it might be associated with a reduced incidence of valvular heart disease, the exact mechanism of which is difficult to explain. Our study is similar to a published MR analysis by Xiao that examined the causal associations of low-density lipoprotein, triglycerides, and high-density lipoprotein with the development of HF and concluded that these lipid components were significantly associated with the development of HF but did not examine the effect of TC on HF [44]. Our study could be a further addition to the literature. Hypoalbuminemia is often recognized as a risk factor for the development of HF and predicts the prognosis of several cardiovascular diseases, including HF [45]. However, we did not find a causal association between serum albumin levels and HF development. Our study also demonstrated that hemoglobin and vitamin D deficiency are not associated with and are not independent risk factors for the development of HF, which is consistent with existing observational studies and consolidates the current evidence.

We found a significant reciprocal causal association between genetically predicted UWP and the onset of HF. There has been early interest in the existence of a relationship between walking and HF, such as the 6-min walk test, which is commonly used in clinical practice, not only to assess the severity of HF but also as a predictor of prognostic judgment [46]. A retrospective study found that changes in gait speed were negatively associated with all-cause mortality from acute HF (per 0.1 m/s increase, HR = 0.83, 95%CI, 0.73–0.95, *P* = 0.006) and with the risk of readmission (HR = 0.91, 95%CI, 0.83–0.99, *P* = 0.036) [47,48]. Another study with a median follow-up time of 16.9 years showed that walking speed was significantly negatively associated with the overall risk of HF in postmenopausal women [49]. In patients with HF aged ≥65 years, walking speeds below 0.527 of the standardized speed were associated with a significant increase in mortality, even after accounting for age- and sex-related decreases in stepping speed [50]. These observational studies were unable to distinguish the causal associations between step speed and HF. Several recently published MR studies have suggested an association between walking speed and the development of HF in terms of genetic predisposition, similar to the findings of our study. However, the published MR analyses did not include reverse MR analyses and failed to reflect the full picture of the causal association between walking speed and HF [51,52]. Unexpectedly, we found a reverse causality between UWP and HF, which persisted even after removing obesity confounders. Higher walking speed helped reduce the risk of HF, and this association may have arisen because of the protective effect of walking speed on hypertension independent of valvular heart disease, cardiomyopathy, and coronary heart disease. The onset of HF can lead to reduced in walking speed. This reciprocal causation is consistent with clinical practice. Furthermore, despite the observational evidence of a strong relationship between grip strength and HF [53], no causal association was observed in the MR analysis.

EA is another important component of the nutritional assessment of patients with HF. Over the past two decades, the association of EA with cardiovascular disease and malnutrition has gradually been emphasized. Although EA is not intuitively related to the functioning of human organs, many observational studies have demonstrated a strong association. The Atherosclerosis Risk in Communities Study (ARIC) focused on assessing the mediating role of the causal pathways of EA and HF. The study, which included 12,109 participants with a median follow-up of 25.1 years, showed a negative association between EA and the risk of HF (HR = 1.41, 95%CI, 1.26–1.57). Mediation analyses revealed that income, waist-to-hip ratio, current smoking, BMI, current drinking, sports, and physical activity mediated the association between EA and HF [54]. The Prospective Urban Rural Epidemiology (PURE) study showed that in the total population, the population-attributable fraction of deaths caused by low EA was the largest, and the harm was even higher than that of smoking. Low EA levels are also closely associated with malnutrition [55]. A systematic review of 34,703 individuals showed that malnutrition and the risk of malnutrition were strongly associated with low EA (OR = 1.48; 95%CI, 1.33–1.64; *P* < 0.001) [56]. Unlike previous analyses based primarily on observational studies, our results from MR analyses may provide more reliable conclusions because MR analyses are not subject to confounders or reverse causation. Our study further confirms the causal association between EA and HF; a higher EA level reduces the incidence of HF without reverse causation, and this association may be mediated by hypertension and coronary heart disease. Wang conducted an MR study of EA and HF; however, after Bonferroni correction, EA was not associated with HF onset. Before Bonferroni correction, the difference remained statistically marginal (*P* = 0.049). These differences may be related to the use of the GWAS database [57].

Our study has some limitations. Although MR is believed to have the advantage of naturally eliminating confounders, some potential and unknown confounders cannot be eliminated, leading to conclusions that need to be viewed with caution. In addition, there may have been other clinically important nutritional assessment phenotypes as well as other unknown mediators of the causal associations that were not included in this study. This should be further analyzed in depth in future studies.

## 5 Conclusions

BMI, WC, and WBFM are potential risk factors for HF, and the correlation between WBFM and HF is significantly stronger than that between BMI and WC, and HF. EA, UWP, and TC are potential protective factors against HF. Common risk factors for HF mediate these causal pathways. Early identification of potential risk or protective factors for HF patients from the dimension of nutritional status is expected to further improve patient outcomes.

## Funding

This study was supported by the "National Mentorship Program" (No. Qngg2022049) and the Jiangsu Province Traditional Chinese Medicine Science and Technology Development Plan General Projects (No. MS2023106).

## Additional information

No additional information is available for this paper.

## Ethics statement

Informed consent was not required for this study because the data for this study were approved by the ethics committee of the original GWASs, and written informed consent was obtained from each participant before data collection.

## Data availability statement

Data will be made available on request.

## CRediT authorship contribution statement

**Yun-Hu Chen:** Writing – review & editing, Writing – original draft, Methodology, Conceptualization. **Mo-Qing Yin:** Validation, Formal analysis. **Li-Hua Fan:** Validation, Formal analysis. **Xue-Chun Jiang:** Investigation, Data curation. **Hong-Feng Xu:** Resources. **Xing-Yu Zhu:** Resources. **Tao Zhang:** Investigation, Data curation.

## Declaration of competing interest

The authors declare that they have no known competing financial interests or personal relationships that could have appeared to influence the work reported in this paper.

## References

[1] Savarese G., Becher P.M., Lund L.H., Seferovic P., Rosano G.M.C., Coats A.J.S. (2023). Global burden of heart failure: a comprehensive and updated review of epidemiology. Cardiovasc. Res..

[2] Dent E., Wright O.R.L., Woo J., Hoogendijk E.O. (2023). Malnutrition in older adults. Lancet (London, England).

[3] Zanetti M., Veronese N., Riso S., Boccardi V., Bolli C., Cintoni M., Francesco V.D., Mazza L., Onfiani G., Zenaro D. (2023). Polypharmacy and malnutrition in older people: a narrative review. Nutrition.

[4] Driggin E., Cohen L.P., Gallagher D., Karmally W., Maddox T., Hummel S.L., Carbone S., Maurer M.S. (2022). Nutrition assessment and dietary interventions in heart failure: JACC review topic of the week. J. Am. Coll. Cardiol..

[5] Vest A.R., Chan M., Deswal A., Givertz M.M., Lekavich C., Lennie T., Litwin S.E., Parsly L., Rodgers J.E., Rich M.W. (2019). Nutrition, obesity, and Cachexia in patients with heart failure: a consensus statement from the heart failure society of America scientific statements committee. J. Card. Fail..

[6] Lin H., Zhang H., Lin Z., Li X., Kong X., Sun G. (2016). Review of nutritional screening and assessment tools and clinical outcomes in heart failure. Heart Fail. Rev..

[7] Sze S., Pellicori P., Zhang J., Weston J., Clark A.L. (2021). The impact of malnutrition on short-term morbidity and mortality in ambulatory patients with heart failure. The American journal of clinical nutrition.

[8] Sze S., Pellicori P., Zhang J., Clark A.L. (2019). Malnutrition, congestion and mortality in ambulatory patients with heart failure. Heart (British Cardiac Society).

[9] Bowden J., Holmes M.V. (2019). Meta-analysis and Mendelian randomization: a review. Res. Synth. Methods.

[10] Birney E. (2022). Mendelian randomization. Cold Spring Harbor perspectives in medicine.

[11] Skrivankova V.W., Richmond R.C., Woolf B.A.R., Yarmolinsky J., Davies N.M., Swanson S.A., VanderWeele T.J., Higgins J.P.T., Timpson N.J., Dimou N. (2021). Strengthening the reporting of observational studies in epidemiology using Mendelian randomization: the STROBE-MR statement. JAMA.

[12] Lee J.J., Wedow R., Okbay A., Kong E., Maghzian O., Zacher M., Nguyen-Viet T.A., Bowers P., Sidorenko J., Karlsson Linnér R. (2018). Gene discovery and polygenic prediction from a genome-wide association study of educational attainment in 1.1 million individuals. Nat. Genet..

[13] Shah S., Henry A., Roselli C., Lin H., Sveinbjörnsson G., Fatemifar G., Hedman Å.K., Wilk J.B., Morley M.P., Chaffin M.D. (2020). Genome-wide association and Mendelian randomisation analysis provide insights into the pathogenesis of heart failure. Nat. Commun..

[14] Codd V., Nelson C.P., Albrecht E., Mangino M., Deelen J., Buxton J.L., Hottenga J.J., Fischer K., Esko T., Surakka I. (2013). Identification of seven loci affecting mean telomere length and their association with disease. Nat. Genet..

[15] Burgess S., Butterworth A., Thompson S.G. (2013). Mendelian randomization analysis with multiple genetic variants using summarized data. Genet. Epidemiol..

[16] Bowden J., Davey Smith G., Haycock P.C., Burgess S. (2016). Consistent estimation in Mendelian randomization with some invalid instruments using a weighted median estimator. Genet. Epidemiol..

[17] Bowden J., Davey Smith G., Burgess S. (2015). Mendelian randomization with invalid instruments: effect estimation and bias detection through Egger regression. Int. J. Epidemiol..

[18] Jia Y., Guo D., Sun L., Shi M., Zhang K., Yang P., Zang Y., Wang Y., Liu F., Zhang Y. (2022). Self-reported daytime napping, daytime sleepiness, and other sleep phenotypes in the development of cardiometabolic diseases: a Mendelian randomization study. European journal of preventive cardiology.

[19] Ong J.S., MacGregor S. (2019). Implementing MR-PRESSO and GCTA-GSMR for pleiotropy assessment in Mendelian randomization studies from a practitioner's perspective. Genet. Epidemiol..

[20] Verbanck M., Chen C.Y., Neale B., Do R. (2018). Detection of widespread horizontal pleiotropy in causal relationships inferred from Mendelian randomization between complex traits and diseases. Nat. Genet..

[21] Yao S., Zhang M., Dong S.S., Wang J.H., Zhang K., Guo J., Guo Y., Yang T.L. (2022). Bidirectional two-sample Mendelian randomization analysis identifies causal associations between relative carbohydrate intake and depression. Nat. Human Behav..

[22] He J., Huang M., Li N., Zha L., Yuan J. (2023). Genetic association and potential mediators between Sarcopenia and coronary heart disease: a bidirectional two-sample, two-step Mendelian randomization study. Nutrients.

[23] Aguilar-Gallardo J.S., Romeo F.J., Bhatia K., Correa A., Mechanick J.I., Contreras J.P. (2022). Severe obesity and heart failure. Am. J. Cardiol..

[24] Sciomer S., Moscucci F., Salvioni E., Marchese G., Bussotti M., Corrà U., Piepoli M.F. (2020). Role of gender, age and BMI in prognosis of heart failure. European journal of preventive cardiology.

[25] Wang Y., Zhang Q., Qi W., Zhang N., Li J., Tse G., Li G., Wu S., Liu T. (2023). Proteinuria, body mass index, and the risk of New-onset heart failure: a prospective cohort study in Northern China. Curr. Probl. Cardiol..

[26] Milajerdi A., Djafarian K., Shab-Bidar S., Speakman J.R. (2018). Pre- and post-diagnosis body mass index and heart failure mortality: a dose-response meta-analysis of observational studies reveals greater risk of being underweight than being overweight. Obes. Rev. : an official journal of the International Association for the Study of Obesity.

[27] Zhou Y., Zha L., Pan S. (2022). The risk of atrial fibrillation increases with Earlier onset of obesity: a Mendelian randomization study. International journal of medical sciences.

[28] Carbone S., Canada J.M., Billingsley H.E., Siddiqui M.S., Elagizi A., Lavie C.J. (2019). Obesity paradox in cardiovascular disease: where do we stand?. Vasc. Health Risk Manag..

[29] Butt J.H., Petrie M.C., Jhund P.S., Sattar N., Desai A.S., Køber L., Rouleau J.L., Swedberg K., Zile M.R., Solomon S.D. (2023). Anthropometric measures and adverse outcomes in heart failure with reduced ejection fraction: revisiting the obesity paradox. Eur. Heart J..

[30] Donataccio M.P., Vanzo A., Bosello O. (2021). Obesity paradox and heart failure. Eat. Weight Disord. : EWD.

[31] Täger T., Franke J., Frey N., Frankenstein L., Fröhlich H. (2023). Prognostic relevance of gradual weight changes on long-term mortality in chronic heart failure. Nutr. Metabol. Cardiovasc. Dis. : Nutr. Metabol. Cardiovasc. Dis..

[32] Holmes C.J., Racette S.B. (2021). The utility of body composition assessment in nutrition and clinical practice: an Overview of current methodology. Nutrients.

[33] Smith L.O., Olieman J.F., Berk K.A., Ligthart-Melis G.C., Earthman C.P. (2023). Clinical applications of body composition and functional status tools for nutrition assessment of hospitalized adults: a systematic review. JPEN - J. Parenter. Enter. Nutr..

[34] Chen Q., Wu Y., Gao Y., Zhang Z., Shi T., Yan B. (2022). Effect of visceral adipose tissue mass on coronary artery disease and heart failure: a Mendelian randomization study. Int. J. Obes..

[35] Sedlmeier A.M., Baumeister S.E., Weber A., Fischer B., Thorand B., Ittermann T., Dörr M., Felix S.B., Völzke H., Peters A. (2021). Relation of body fat mass and fat-free mass to total mortality: results from 7 prospective cohort studies. The American journal of clinical nutrition.

[36] Kulyté A., Lundbäck V., Arner P., Strawbridge R.J., Dahlman I. (2022). Shared genetic loci for body fat storage and adipocyte lipolysis in humans. Sci. Rep..

[37] Paixão da Silva E., Ranielly Dos Santos Avelino R., Zuza Diniz R.V., Dantas de Lira N.R., Monteiro Lourenço Queiroz S.I., Gomes Dantas Lopes MM., Maurício Sena-Evangelista K.C. (2023). Body composition, lipid profile and clinical parameters are predictors of prognosis in patients with heart failure: two-year follow-up. Clinical nutrition ESPEN.

[38] Aune D., Sen A., Norat T., Janszky I., Romundstad P., Tonstad S., Vatten L.J. (2016). Body mass index, Abdominal Fatness, and heart failure incidence and mortality: a systematic review and dose-response meta-analysis of prospective studies. Circulation.

[39] Zhou R., Yang M., Yue C., Shi Y., Tan Y., Zha L., Zhang J., Chen S. (2023). Association between dietary choline intake and cardiovascular diseases: National health and nutrition Examination survey 2011-2016. Nutrients.

[40] Halldin A.K., Lissner L., Lernfelt B., Björkelund C. (2020). Cholesterol and triglyceride levels in midlife and risk of heart failure in women, a longitudinal study: the prospective population study of women in Gothenburg. BMJ Open.

[41] Arafa A., Kashima R., Kokubo Y., Teramoto M., Sakai Y., Nosaka S., Kawachi H., Shimamoto K., Matsumoto C., Nakao Y.M. (2023). Serum cholesterol levels and the risk of brain natriuretic peptide-diagnosed heart failure in postmenopausal women: a population-based prospective cohort study. Menopause.

[42] Cunha F.M., Pereira J., Ribeiro A., Silva S., Araújo J.P., Leite-Moreira A., Bettencourt P., Lourenço P. (2019). The cholesterol paradox may be attenuated in heart failure patients with diabetes. Minerva Med..

[43] Wang B., Liu J., Chen S., Ying M., Chen G., Liu L., Lun Z., Li H., Huang H., Li Q. (2021). Malnutrition affects cholesterol paradox in coronary artery disease: a 41,229 Chinese cohort study. Lipids Health Dis..

[44] Xiao J., Ji J., Zhang N., Yang X., Chen K., Chen L., Huang W. (2023). Association of genetically predicted lipid traits and lipid-modifying targets with heart failure. European journal of preventive cardiology.

[45] Gopal D.M., Kalogeropoulos A.P., Georgiopoulou V.V., Tang W.W., Methvin A., Smith A.L., Bauer D.C., Newman A.B., Kim L., Harris T.B. (2010). Serum albumin concentration and heart failure risk the health, aging, and body composition study. Am. Heart J..

[46] Ferreira J.P., Metra M., Anker S.D., Dickstein K., Lang C.C., Ng L., Samani N.J., Cleland J.G., van Veldhuisen D.J., Voors A.A. (2019). Clinical correlates and outcome associated with changes in 6-minute walking distance in patients with heart failure: findings from the BIOSTAT-CHF study. Eur. J. Heart Fail..

[47] Tanaka S., Kamiya K., Hamazaki N., Matsuzawa R., Nozaki K., Nakamura T., Yamashita M., Maekawa E., Noda C., Yamaoka-Tojo M. (2019). Short-term change in gait speed and clinical outcomes in older patients with acute heart failure. Circ. J. : official journal of the Japanese Circulation Society.

[48] Imran T.F., Orkaby A., Chen J., Selvaraj S., Driver J.A., Gaziano J.M., Djoussé L. (2019). Walking pace is inversely associated with risk of death and cardiovascular disease: the Physicians' Health Study. Atherosclerosis.

[49] Miremad M.M., Lin X., Rasla S., El Meligy A., Roberts M.B., Laddu D., Allison M., Martin L.W., Shadyab A.H., Manson J.A.E. (2022). The association of walking pace and incident heart failure and subtypes among postmenopausal women. J. Am. Geriatr. Soc..

[50] Ozawa T., Yamashita M., Seino S., Kamiya K., Kagiyama N., Konishi M., Saito H., Saito K., Ogasahara Y., Maekawa E. (2021). Standardized gait speed ratio in elderly patients with heart failure. ESC heart failure.

[51] Chen L., Sun X., He Y., Zheng L. (2022). Self-reported walking pace and risk of cardiovascular diseases: a two-sample Mendelian randomization study. Front. Genet..

[52] Timmins I.R., Zaccardi F., Nelson C.P., Franks P.W., Yates T., Dudbridge F. (2020). Genome-wide association study of self-reported walking pace suggests beneficial effects of brisk walking on health and survival. Commun. Biol..

[53] Parahiba S.M., Spillere S.R., Zuchinali P., Padilha G.D.R., Duarte M.B., da Silveira I.V., Dias L.H., Knobloch I.D.S., Perry I.S., Souza G.C. (2021). Handgrip strength in patients with acute decompensated heart failure: accuracy as a predictor of malnutrition and prognostic value. Nutrition.

[54] Lin Y., Zhang S., Wang S., Zhong X., Li Y., Xiong Z., Sun X., Huang Y., Fan Y., Guo Y. (2021). Behavioral factors mediating the impact of educational attainment on incident heart failure - a mediation analysis. Circ. J. : official journal of the Japanese Circulation Society.

[55] Yusuf S., Joseph P., Rangarajan S., Islam S., Mente A., Hystad P., Brauer M., Kutty V.R., Gupta R., Wielgosz A. (2020). Modifiable risk factors, cardiovascular disease, and mortality in 155 722 individuals from 21 high-income, middle-income, and low-income countries (PURE): a prospective cohort study. Lancet (London, England).

[56] Besora-Moreno M., Llauradó E., Tarro L., Solà R. (2020). Social and economic factors and malnutrition or the risk of malnutrition in the elderly: a systematic review and meta-analysis of observational studies. Nutrients.

[57] Wang W., Wang J., Zhuang Z., Gao M., Yang R., Liu Z., Huang T. (2021). Assessment of causality between modifiable factors and heart failure: a Mendelian randomization analysis. Asia Pac. J. Clin. Nutr..

